The article "Multichannel Saliency Detection Based on Visual Bionics" was published in 2020. Journal: Appl Bionics Biomech.

# Multichannel Saliency Detection Based on Visual Bionics

**DOI:** 10.1155/2020/8886923

**Published:** 2020-11-23

**Authors:** Lidan Cheng, Tianyi Li, Shijia Zha, Wei Wei, Jihua Gu

**Affiliations:** College of Optoelectronics Science and Engineering, Soochow University, Suzhou Jiangsu Province 215000, China

## Abstract

Inspired by the visual properties of the human eyes, the depth information of visual attention is integrated into the saliency detection to effectively solve problems such as low accuracy and poor stability under similar or complex background interference. Firstly, the improved SLIC algorithm was used to segment and cluster the RGBD image. Secondly, the depth saliency of the image region was obtained according to the anisotropic center-surround difference method. Then, the global feature saliency of RGB image was calculated according to the colour perception rule of human vision. The obtained multichannel saliency maps were weighted and fused based on information entropy to highlighting the target area and get the final detection results. The proposed method works within a complexity of O(N), and the experimental results show that our algorithm based on visual bionics effectively suppress the interference of similar or complex background and has high accuracy and stability.

## 1. Introduction

Saliency detection is an important research content in computer vision, which refers to the process of simulating human visual attention mechanism to accurately and quickly detect the most interesting regions in images. Borji et al. defined that saliency visually described the prominent target or area in the scene relative to its neighbouring area [1]. The human visual attention mechanism prioritizes a few significant areas or objectives, while ignoring or discarding others that are not, which can allocate computing resources selectively and greatly improve the efficiency of visual information processing. Therefore, the saliency computing model based on visual attention mechanism has been widely studied. When processing the input image or video, the computer can judge the importance of its visual information by detecting the saliency area. It has been widely applied in object detection and identification [2], image retrieval [3], video quality assessment [4], video compression [5], image cropping [6], and other fields.

The RGB image saliency detection model based on visual attention mechanism uses low-level feature contrast to calculate saliency [7, 8]. Typical of them are global feature comparison calculation model [9], local feature comparison calculation model [10], and combination of global and local feature comparison model [11]. In order to improve the accuracy of detection, the saliency detection model was proposed based on prior knowledge [12]. Typical of them are position prior [13], background prior [14, 15], colour prior [16], shape prior [17], and boundary prior [18, 19].

The article "Multichannel Saliency Detection Based on Visual Bionics" was published in 2020. Journal: Appl Bionics Biomech.

However, most 2D image saliency detection models based on human visual attention mechanism ignore the fact that human visual attention mechanism is based on 3D scene. It shows that depth provides extra important information of saliency detection for RGB image. Desingh et al. discussed 3D saliency detection methods based on depth appearance, depth-induced blur, and centre-bias [20]. Niu et al. conducted depth saliency detection based on parallax contrast and professional knowledge in vertical photography [21]. Further, Ju et al. proposed a depth saliency detection model based on depth image anisotropic center-surround difference [22]. Ren et al. [23], respectively, proposed the saliency detection of RGB-D images against a complex background by combining the prior knowledge of depth, indicating the validity of depth information in 3D saliency detection. However, there are two challenges in the process of saliency detection of RGB-D images. The first is how to calculate the saliency of depth images under similar or complex background interference, and the second is how to combine the saliency map of depth image and RGB image to obtain the final result with a good performance. In this paper, we proposed a multichannel saliency detection method based on RGBD images, which has the following contributions:

1. On the basis of SLIC algorithm, colour, texture, and depth information are used to measure the distance of superpixel segmentation
2. Based on the perception rule of human vision, we introduced the depth information and global information of RGB image as two feature channels for saliency computing
3. The weighted features of depth saliency and colour saliency were fused by information entropy, and experiment shows that the algorithm has a good performance in case of background interference

## 2. Saliency Detection

The algorithm framework of this paper is shown in Figure 1. Combining the depth map with the RGB map to carry out image preprocessing and colour, texture, and depth information are introduced as the basis of superpixel segmentation. Then, the colour and depth information were calculated as two feature channels of saliency map. As is shown in Figure 2, the depth saliency was obtained by the anisotropic center-surround difference (ACSD) method, and the global saliency of RGB image was calculated by global contrast method based on HSV space. Finally, information entropy is used to calculate the weights of two channels, respectively, and get the final fused saliency map.

The article "Multichannel Saliency Detection Based on Visual Bionics" was published in 2020. Journal: Appl Bionics Biomech.

## 3. Image Preprocessing

The human visual observation system takes the image region as the basic unit, and the saliency detection based on the region conforms to the visual characteristics of the human eyes. As a construction method of pixel region, superpixel technology has been widely used in computer vision field. Superpixel can quickly segment the image into subregions with certain semantics, which is conducive to the extraction of local features and the expression of structural information [24]. SLIC algorithm has obtained a good balance in the two aspects of edge fitting degree and compactness, which has an excellent comprehensive performance. When the SLIC is used to segment the left image, the obtained boundary is not accurate because of ignoring the mutual constraint relationship between the 2D and depth information. Therefore, colour, texture, and depth information are used to measure the distance of superpixel segmentation in this paper.

Converting the left image to the CIE Lab colour space and dividing the image into *k* superpixels. Here, each pixel has a unique identifier  *i*. Extract the follow 7 d characteristics of each superpixel region as measurement property. It can be expressed:

(1) $$\begin{array}{c} S_{p¯i}=\left\{l_{i},a_{i},b_{i},C_{\text{con}i},C_{\text{cor}i},E_{i},d_{i}\right\}\;i=1,2,3,\cdots ,k, \end{array}$$

where *l*_*i*_, *a*_*i*_, and *b*_*i*_ are the mean value of *L*, *a*, and *b* colour components of each superpixel region; *C*_con*i*_, *C*_cor*i*_, and *E*_*i*_  are the mean value of contrast, cross-correlation, and energy mean of gray level cooccurrence matrix of each superpixel region; and *d*_*i*_ is the depth value of each superpixel region. Then, we can describe the adjacent superpixel pair as *S*_*p*¯*ij*_:

(2) $$\begin{array}{c} S_{p¯ij}=\left\{\left(S_{p¯i},S_{p¯j}\right)\right\}\;i\in \left[1,k\right],j\in \left[1,k\right],i\neq j, \end{array}$$

where *S*_*p*¯*ij*_ superpixel pair with *i* and *j* as identifier, *k* is the number of superpixels of the image, and *S*_*P*¯*i*_ and *S*_*p*¯*j*_ are the 7 d characteristics of the adjacent superpixel pair. The number of adjacent superpixel pairs in each image is determined by SLIC superpixel segmentation.

Using colour, texture, and depth features to calculate the difference between all adjacent superpixel pairs *S*_*p*¯*ij*_.  *d*_*lab*_, *d*_*glcm*_, and *d*_depth_ are defined to describe the measurement of colour, texture and depth characters:

(3) $$\begin{array}{c} d_{lab}=\sqrt{{\left(l_{i}-l_{j}\right)}^{2}+{\left(a_{i}-a_{j}\right)}^{2}+{\left(b_{i}-b_{j}\right)}^{2},}\\ \;d_{glcm}=\sqrt{{\left(C_{\text{con}i}-C_{\text{con}j}\right)}^{2}+{\left(C_{\text{cor}i}-C_{\text{cor}j}\right)}^{2}+{\left(E_{i}-E_{j}\right)}^{2},}\\ \;d_{\text{depth}}=\sqrt{\;{\left(d_{i}-d_{j}\right)}^{2}.} \end{array}$$

Then, the distance measurement of superpixel segmentation *D*_*ij*_ is

(4) $$\begin{array}{c} D_{ij}=\omega_{1}∙\sqrt{\frac{\varepsilon +d_{lab}^{2}}{3}}+\omega_{2}∙\sqrt{\frac{\varepsilon +d_{glcm}^{2}}{3}}+\omega_{3}∙\sqrt{\varepsilon +d_{\text{depth}}^{2}}, \end{array}$$

where *ε* = 10^−4^. It is used to ensure the validity of the value. *ω*_1_, *ω*_2_, are *ω*_3_ are the weight of colour, texture, and depth.

The article "Multichannel Saliency Detection Based on Visual Bionics" was published in 2020. Journal: Appl Bionics Biomech.

In the image, the greater the discreteness of a feature data set is, it means that the more influence this feature has on the image. Mean variance can effectively represent the degree of difference between data. Therefore, the global mean variance of colour, texture, and depth is used as the weight values of the three features *ω*_1_, *ω*_2_, and *ω*_3_.

If the difference between adjacent superpixels is less than a certain threshold th_1_, the adjacent superpixel pair will be merged.

(5) $$\begin{array}{c} {\text{th}}_{1}=\sqrt{\frac{\omega_{1}∙\left(\bar{l}+\bar{a}+\bar{b}\right)}{3}}+\sqrt{\frac{\omega_{2}∙\left(\bar{C_{\text{con}}}+\bar{C_{\text{cor}}}+\bar{E}\right)}{3}}+\sqrt{\omega_{3}∙\bar{d}}, \end{array}$$

where $\bar{l},\bar{a},$ and $\bar{b}$ are the mean value of *L*, *a*, and *b* colour components of the image; $\bar{C_{\text{con}}},\bar{C_{\text{cor}}},$ and $\bar{E}$ are the mean value of contrast, cross-correlation, and energy mean of gray level cooccurrence matrix of the image; and $\bar{d}$ is the depth value of the image.

Finding all similar adjacent superpixel pairs and taking the upper left superpixel of the image as the starting point of clustering. The output after clustering contains *n* regions *R*_*i*_, 1 ≤ *i* ≤ *n*.

## 4. Depth Saliency Map

For each superpixel, the anisotropic center-surround difference (ACSD) value is calculated, and the value of center superpixel is assigned to each pixel within the region *R*_*i*_. Performing an anisotropic scan along multiple directions, in each scanline, assuming the pixel with the minimum depth value as background and calculate the difference between the center pixel and background. *L* is the maximum scan length for each scanline. The typical value of *L* is a third of the diagonal length.

The anisotropic center-surround difference (ACSD) is summed over eight scanning directions 0°, 45°, 90°, 135°, 180°, 225°, 270°, and 315°. The mathematical description of anisotropic center-surround difference (ACSD) measure is

(6) $$\begin{array}{c} S_{d}^{m}\left(x,y\right)=d\left(x,y\right)-\min\left(d^{m}\right),n\in \left[1,L\right],\\ S_{d}\left(x,y\right)=\overset{8}{\underset{m=1}{\sum }}S_{d}^{m}, \end{array}$$

where *S*_depth_^*m*^ indicates the ACSD value of pixel (*x*, *y*) along the scanline *m*. *d*(*x*, *y*) is the depth value of pixel (*x*, *y*). *n* is the index of the pixels along the scan path *m*. min(*d*^*m*^) is the minimum depth value along the scanline *m*. *S*_*d*_(*x*, *y*) is the ACSD value of pixel (*x*, *y*) which sums the center-surround difference values in eight directions.

The article "Multichannel Saliency Detection Based on Visual Bionics" was published in 2020. Journal: Appl Bionics Biomech.

## 5. Global Saliency Map of RGB Image

Colour histogram is used to regularize the colour of the image to level 128 in order to reduce the computational complexity and save the storage space. On the other hand, the descending dimension algorithm for HSV colour space is proposed. With the decrease of saturation, any colour in HSV space can be described by the change of gray level. The intensity value determines the specific gray level of the conversion [25]. When the colour saturation is close to zero, all pixels look similar regardless of hue. With the increase of saturation, the pixels are distinguished by hue value.

Compared with colour saturation, human vision is more sensitive to hue and intensity. The pixels with lower colour saturation can be approximately represented by intensity level, while the pixels with higher colour saturation can be approximately represented by hue. Saturation value is used to determine whether each pixel can be represented by hue or intensity value, which is more consistent with the law of human visual perception. Saturation threshold th_2_ is

(7) $$\begin{array}{c} {\text{th}}_{2}=1-\frac{0.8\;I_{v}\left(x,y\right)}{255}, \end{array}$$

where *I*_*v*_(*x*, *y*) represents the *V* component value of a pixel. When the saturation value *I*_*s*_(*x*, *y*) is greater than th_2_, the pixel point is represented by the hue value *I*_*v*_(*x*, *y*); when the saturation value is less than th_2_, the pixel point is represented by the intensity value *I*_*h*_(*x*, *y*). The saliency of each pixel is

(8) $$\begin{array}{c} S_{c}\left(x,y\right)=\left\{\begin{array}{c} \left|\bar{I}-I_{v}\left(x,y\right)\right|\;I_{s}\left(x,y\right)\leq {\text{th}}_{2}\\ \left|\bar{I}-I_{h}\left(x,y\right)\right|\;I_{s}\left(x,y\right)>{\text{th}}_{2} \end{array}\right.\forall \left(x,y\right)\in R_{i}, \end{array}$$

where *I*_*s*_(*x*, *y*)  is the saturation value of the pixel, *I*_*h*_(*x*, *y*)  is the hue value of the pixel, *I*_*v*_(*x*, *y*) is the intensity value of the pixel, and $\bar{I}$ is the mean value of all pixels.

## 6. Fusion of Saliency Map

When synthesizing the colour saliency map and the depth saliency map, the information entropy is used to calculate the weights of the channels.

The article "Multichannel Saliency Detection Based on Visual Bionics" was published in 2020. Journal: Appl Bionics Biomech.

The information entropy of colour saliency is

(9) $$\begin{array}{c} H_{c}\left(R\right)=-\overset{n}{\underset{i=1}{\sum }}p_{c}\left(R_{i}\right)\log\left(p_{c}\left(R_{i}\right)\right), \end{array}$$

where *p*_*c*_(*R*_*i*_) is the ratio of the sum of *R*_*i*_ colour saliency values to the whole image.

The information entropy of depth saliency is

(10) $$\begin{array}{c} H_{d}\left(R\right)=-\overset{n}{\underset{i=1}{\sum }}p_{d}\left(R_{i}\right)\log\left(p_{d}\left(R_{i}\right)\right), \end{array}$$

where *p*_*d*_(*R*_*i*_) is the ratio of the sum of  *R*_*i*_ depth saliency values of to the whole image.

The saliency map *S*_fuse_(*x*, *y*) was obtained by fusing the two channels:

(11) $$\begin{array}{c} S_{\text{fuse}}\left(x,y\right)=\frac{H_{c}\left(R\right)}{H_{c}\left(R\right)+H_{d}\left(R\right)}S_{c}\left(x,y\right)+\frac{H_{d}\left(R\right)}{H_{c}\left(R\right)+H_{d}\left(R\right)}S_{d}\left(x,y\right)\forall \left(x,y\right)\in R_{i}. \end{array}$$

## 7. Experimental Comparison

We show a few saliency maps generated by different algorithms in Figure 3.

The precision-recall curve is evaluated from two aspects: precision and recall. Precision refers to the ratio between the number of correct saliency pixels and the whole number of saliency pixels, which is used as the *y*-axis. Recall refers to the ratio of the number of correct saliency pixels to the number of true pixels, which is used as the *x*-axis.

The algorithms are tested on NJU400 datasets. Two test sets are divided from NJU400 according to the complexity and the similarity of the background. Four volunteers are invited to divide the raw datasets into the normal group (N group) and the similar/complex background group (S/C group). At last, 92 high quality and consistently labelled images are selected into the S/C group, and the rest are divided into the N group. The precision-recall curves of different algorithms tested on the N group, S/C group, and full datasets are given in Figure 4. The performance of different algorithms tested on three groups is given in Table 1.

The proposed method works within a complexity of O(N), and the evaluation on the results of these saliency detection algorithms in the S/C group shows that our algorithm has a better performance than other algorithms. In full datasets, it also performs well. By selecting the salient subset for further processing, the complexity of higher visual analysis can be reduced significantly. Many applications benefit from saliency analysis such as object segmentation, image classification, and image/video retargeting.

The article "Multichannel Saliency Detection Based on Visual Bionics" was published in 2020. Journal: Appl Bionics Biomech.

## 8. Conclusions

A new framework based on visual bionics for saliency detection under similar or complex background interference is proposed in this paper: First, we combine the depth map with the RGB map, and colour, texture, and depth information are introduced as the basis of superpixel segmentation. Second, the colour and depth information were calculated as two feature channels of saliency map. Finally, information entropy is used to calculate the weights of two channels, respectively, and get the final fused saliency map. The proposed method works within a complexity of O(N), and the experimental results show that our saliency detection framework greatly reduces the error detection under similar and complex background and improves the overall saliency detection performance.

## Figures and Tables

**Figure 1:** Our framework of saliency detection.

**Figure 2:** Example of the ACSD operator in a region.

**Figure 3:** Saliency comparisons of different methods in terms of NJU400 dataset: (a) RGB image; (b) depth image; (c) ground truth; (d) GS; (e) MC; (f) MR; (g) WCTR; (h) ACSD; (i) MSD.

**Figure 4:** The precision-recall curves of different algorithms: (a) the precision-recall curves on the N group; (b) the precision-recall curves on the S/C group; (c) the precision-recall curves on full datasets.

**Table 1:** The performance of different algorithms tested on three groups.

Group	Algorithms	Precision
N group	GS	0.68
	MC	0.79
	MR	0.85
	RBD	0.81
	ACSD	0.84
	MSD	0.82

S/C group	GS	0.49
	MC	0.50
	MR	0.63
	RBD	0.56
	ACSD	0.87
	MSD	0.95

Full datasets	GS	0.64
	MC	0.72
	MR	0.80
	RBD	0.76
	ACSD	0.81
	MSD	0.86

## Data Availability

The NJU400 datasets used to support the findings of this study are included within the article.
